# Design of International Chinese Education Promotion Platform Based on Artificial Intelligence and Facial Recognition Technology

**DOI:** 10.1155/2022/6424984

**Published:** 2022-07-13

**Authors:** Yi Shen, Sixian Sun

**Affiliations:** ^1^Southwest University, Beibei, Chongqing 400715, China; ^2^Yunnan Normal University, Kunming, Yunnan 650092, China; ^3^Chiang Rai Rajabhat University, Chiang Rai 57100, Thailand; ^4^Primary School Attached to Yunnan Normal University, Kunming, Yunnan 650031, China

## Abstract

With the continuous development of today's society, digital image processing technology has been applied in more and more fields, among which authentication in digital image processing technology has become a hot field. In the process of identity verification, the face is used as the basis of feature recognition because the method of using the face as a feature basis is more easily accepted by the public and the operation is simple and the feasibility is stronger. In the online education model, observing and comparing students' facial emotions through the platform and analyzing students' learning goals, learning effects, learning emotions, and contradictions and conflicts arising in the process of cooperation have become an effective teaching evaluation system. Up to now, China has developed into the second largest economy in the world. The global “Chinese fever” has brought China's culture into a new stage of development. Countries in the world learn Chinese culture by developing Chinese language courses. By building a Chinese learning intelligent system with a B/S structure, this system can effectively evaluate the teaching process. It can be seen from the test results that the platform meets the basic requirements of functional design.

## 1. Introduction

Biological characteristics have become the most ideal basis for identity verification due to their stability and individual differences [1]. Among them, using facial features for recognition is the simplest way, and it is easier to be accepted by the majority of users [2]. In the traditional hardware design process, the general-purpose computer systems are used, but the general-purpose computer system has an obvious shortcoming of high-power consumption and low reliability [3]. With the continuous upgrading of technology, new computer systems have gradually developed. Embedded systems have gradually developed into the most commonly used computer systems in today's society due to their high-cost performance, strong real-time performance, and simultaneous operation of multiple tasks. And with the continuous update of embedded systems, its footprint is getting smaller and smaller. At the same time, embedded systems can flexibly formulate processing tasks according to user needs. Therefore, the embedded system has gradually developed into a new force in the current era by virtue of its powerful functions and easy portability [4].

With the continuous development of society, the learning model that combines online learning and offline learning has become the mainstream of today's society. Online learning will not be restricted by objective factors such as time and location, as long as it is connected to the Internet through a mobile device terminal. Online learning can be done, so it is more convenient than offline learning [5]. However, there are still many problems in online learning that need to be solved urgently, such as how to determine the identity of online learners, how to detect the learning effects of learners, and how to conduct teaching feedback with learners [6]. In the process of researching the above problems, this paper divides the research into three aspects: learner face recognition, eye state detection, and emotion perception. In the process of research, learners are comprehensively evaluated and analyzed, and learners' in-depth perception of learning behavior provides new ideas and methods for online learning behavior evaluation through the above methods [7]. At the same time, through comprehensive evaluation and analysis of learners, learners can conduct self-supervision and comprehensiveness in the learning process. Evaluation and analysis can also be used as an external supervisory means for auxiliary supervision [8]. Among the autonomous learning systems supported by computers, CSAL is the main method adopted by today's teaching systems. The CSAL method is based on computer technology and network technology to build a teaching platform. Through this platform, teachers and students can exchange information and share resources. The CSAL method is conducive to the formation of a student-led teaching model. However, the current CSAL teaching system still has certain shortcomings. For example, the CSAL system is still teaching based on forums, and in the teaching process, the teacher's supervision is not strong enough, the learners' consciousness is not high, and the teaching effect is bad. Aiming at the problems of the above CSAL system, this article researches on the working mechanism of CSAL and discusses the theoretical research significance and practical value of the autonomous learning platform. Based on the monitoring results of the learner's learning status, the learner's self-learning effect is analyzed to timely solve the problems of the learner in the process of autonomous learning and actively remind and correct the learner's learning process.

## 2. Related Work

Since entering the end of the 20th century, China's economy has entered a stage of rapid development. Up to now, China has developed into the second largest economy in the world. At the same time, China's influence and status in the international arena are constantly improving. The rise of China has set off a phenomenon of “Chinese fever” around the world [9]. The literature and internet databases are consulted, and various resources are collected and integrated during the consultative process, and the relevant policy materials for Chinese language education in various countries are summarized to facilitate the use in future research [10]. The literature believes that, with the rapid development of science and technology in China, a new era of combining artificial intelligence and education is coming [11]. The relevant content in the literature pointed out that, under the background of today's society, people pay more and more attention to the citation of artificial intelligence technology in the education industry, and according to the relevant content in the article, one of the development trends of future education technology is combined with artificial intelligence technology [12]. Literature studied the “preliminary artificial intelligence” elective module that appeared in the information technology discipline for the first time [13]. The emergence of the “preliminary artificial intelligence” elective module marked that China's artificial intelligence education has entered a new stage of development. A literature believes that, in 2017, China's artificial intelligence education once again ushered in a historical turning point [14]. The relevant content in the literature shows that relevant domestic experts suggest adding courses related to the field of artificial intelligence in primary and secondary schools [15]. At the same time, algorithm programming education should also be promoted in primary and secondary education to continuously improve China's artificial functional disciplines. Continuously improve the quality of artificial intelligence talents in my country. The relevant content in the literature shows that artificial intelligence education has gradually risen from the social level to the national strategic level [16]. Artificial intelligence has gradually become an important indicator to measure the comprehensive competitiveness of the country in the new era, and artificial intelligence has gradually become the main theme of technological development in the 21st century.

## 3. Artificial Intelligence

### 3.1. Research Status

Up to now, with the support of economic conditions, artificial intelligence technology has developed steadily and efficiently for more than 60 years, and the related research results of artificial intelligence technology have gradually become more colorful than before. But if artificial intelligence technology is compared with the history of human science and technology, artificial intelligence technology is still in a preliminary stage of development. At the same time, our humans' philosophical reflection on artificial intelligence is not mature enough, which leads to a series of problems. Therefore, we must first analyze and understand the relevant books on the philosophy of artificial intelligence and then summarize the current research status of artificial intelligence ethics. In recent years, with the continuous innovation of science and technology, the deep learning method based on the artificial neural networks has brought a new wave of development to the development of artificial intelligence. Different learning models, learning methods, and algorithms are comprehensively compared, and the differences in machine learning are studied (Table 1).

The further in-depth research on machine learning has also greatly promoted its application in education.

### 3.2. Natural Language Understanding

With the continuous acceleration of the social process, the research on natural language has gradually developed. The study of understanding natural language is the study of how to make computers understand and generate human language. In the process of studying and understanding natural language, scientists divide natural language into sound language and written language. In the research process, the two parts are separated for research. When understanding natural language, it is necessary to first express the natural language to be understood in a mathematical form, then convert the mathematical form into an algorithm, and finally write a program based on the algorithm. The process is shown in Figure 1.

Natural language understanding technology has developed from the initial production system and rule system to the current statistical model and machine learning methods.

### 3.3. Key Technologies of the Face Recognition System

Artificial neural networks entered a new stage of development about forty years ago, and after a period of rapid development and continuous upgrading, artificial neural networks have gradually become a popular direction in the field of artificial intelligence. The artificial neural network simulates the neural network of the human brain, abstracts the input information, generates a simple model of the processed information, matches the input information with the model, and forms an artificial neural network through a variety of connection methods.

The artificial neural network is composed of the most basic neurons, and the structure of the artificial neural network can be established by connecting multiple simple models of neurons as shown in Figure 1. At the same time, the neuron model can be expressed as

(1) $$\begin{array}{c} y=f\left(\sum_{i=1}^{n}w_{i}x_{i}-\theta \right). \end{array}$$

In the process of interpreting the artificial neural network, the activation function introduces the concept of nonlinear characteristics into the artificial neural network. In the process of screening multiple excitation function forms, it is found that the most matching function model is the unit step function model. However, in the actual application process, since the unit step function is a discontinuous function, the log probability function is usually an excitation function, and it replaces the unit step function model.

The expression of the function is

(2) $$\begin{array}{c} y=\frac{1}{1+e^{-x}}. \end{array}$$

From the image, the output value of the log probability function is between 0 and 1, and the slope of the log probability function is the largest when the output value is 0. Through the analysis of the image, it can also be found that the logarithmic probability function can be derived in any order.

Figure 2 shows the working structure diagram of the most common artificial neural network. The artificial neural network that works with this structure is usually called a multilayer feedforward neural network.

In a multilayer feedforward neural network, the neurons in the previous layer are often connected to the neurons in the next layer one by one, but the neurons in the same layer are not connected in pairs, and two layers that are not adjacent the same are true for neurons. The external signal will first be transmitted from the input layer neurons to the hidden layer neurons, and after processing, finally output by the output layer neurons. To describe the input example, first, input the attribute for corresponding processing, then output the *Y* real-valued vector training set, and then input the obtained training set into the multilayer feedforward neural network. After the hidden layer neuron processing, the output value of the neuron output and the input value received by the neuron of the output layer are

(3) $$\begin{array}{c} \alpha_{h}=\sum_{i=1}^{d}v_{ih}x_{i}, \end{array}$$

(4) $$\begin{array}{c} \beta_{n}=\sum_{h=1}^{q}w_{hn}b_{h}. \end{array}$$

Among them, the connection weight between the input layer neuron and the hidden layer neuron is *T*7*ih*, and the connection weight between the hidden layer and the output layer neuron is *W*_*h*_, assuming that the output result of the output layer is

(5) $$\begin{array}{c} {\hat{y}}_{k}=\left({\hat{y}}_{1}^{k},{\hat{y}}_{1}^{k},\ldots ,{\hat{y}}_{j}^{k}\right), \end{array}$$

(6) $$\begin{array}{c} y_{n}^{k}=f\left(\beta_{n}-\theta_{n}\right). \end{array}$$

Among them, the mean square error of the neural network when outputing the result is

(7) $$\begin{array}{c} E_{k}=\frac{1}{2}\sum_{n=1}^{j}{\left(y_{n}^{k}-{\hat{y}}_{n}^{k}\right)}^{2}, \end{array}$$

(8) $$\begin{array}{c} \Delta W_{hn}=-\eta \frac{\partial E_{k}}{\partial w_{hn}}. \end{array}$$

According to the chain derivation rule, formula (8) can be written as

(9) $$\begin{array}{c} \Delta w_{hn}=-\eta \frac{\partial E_{k}}{\partial {\overset{⌢}{y}}_{n}^{k}}\frac{\partial {\overset{⌢}{y}}_{n}^{k}}{\partial \beta_{n}}\frac{\partial \beta_{n}}{\partial w_{hn}}. \end{array}$$

According to formula (4), we can get

(10) $$\begin{array}{c} \frac{\partial \beta_{n}}{\partial w_{hn}}=b_{h}. \end{array}$$

Change the log probability function to the correlation function of the original function, namely,

(11) $$\begin{array}{c} f^{\prime }=f\left(1-f\right). \end{array}$$

Then, it can be obtained according to equations (6) and (7):

(12) $$\begin{array}{c} g_{n}=\frac{\partial E_{k}}{\partial {\overset{⌢}{y}}_{n}^{k}}\frac{\partial {\overset{⌢}{y}}_{n}^{k}}{\partial \beta_{n}},\\ ={\overset{⌢}{y}}_{n}^{k}\left(1-{\overset{⌢}{y}}_{n}^{k}\right)\left(y_{n}^{k}-{\hat{y}}_{n}^{k}\right). \end{array}$$

Substitute formulas (10) and (12) into formula (9), substitute the result obtained into equation (8), and then use the backpropagation algorithm to calculate the final result:

(13) $$\begin{array}{c} \Delta w_{hn}=\eta g_{n}b_{n}. \end{array}$$

*ne* in the formula represents the learning rate. Each iteration of the learning rate will update the step size in the algorithm. The step size can determine the convergence speed of the formula to a certain extent. By adjusting formula (13), the following new formula is obtained:

(14) $$\begin{array}{c} w_{hn}\leftarrow w_{hn}+\Delta w_{hn}. \end{array}$$

Through observation and analysis at the theoretical level, we can find that there is a certain degree of positive correlation between model parameters and model difficulty. The difficulty of model training is mainly reflected in the long time and high complexity. However, the more parameters of the model do not mean that there is no advantage at all; on the contrary, it has great advantages. The increase of model parameters can greatly enhance the learning ability of the model, enabling it to learn more comprehensively and deeply about those complex data. With the advent of the information age and the development of big data, computing capabilities have been greatly improved, especially in terms of graphics processing unit capabilities, which makes the abovementioned difficulties and problems solved to a large extent. For example, the large amount of training data obtained during the training process greatly reduces the risk of falling into an overfitting state, and the powerful computing power of the graphics processing unit improves the training efficiency. Various advantages have caused people to shift their attention to various complex learning models, especially deep learning. Deep neural networks are representative of deep learning models. Increasing the number of hidden layer neurons can improve the autonomous learning ability of artificial neural networks to a certain extent. Convolutional neural network model is shown in Figure 3.

Not only that, deep learning can also perform feature learning, that is, automatically extracting features from input data. The main process of feature learning is as follows: by using the convolutional neural network in deep learning, the input information is processed based on multiple hidden layers, the original low-level features are gradually transformed into high-level features, and the obtained features are analyzed using simple models. Perform integration or classification, and finally complete the feature learning task. Feature learning not only enhances the quality of the obtained features but also improves the ability to efficiently and smoothly complete real-life tasks through machine learning.

The convolution operation is used in this process. The feature map of the previous layer is first subjected to convolution operation, and then the convolution operation is combined, and finally a corresponding excitation function can be obtained, as follows.

(15) $$\begin{array}{c} x_{j}^{l}=f\left(\sum_{i\in M_{j}}x_{i}^{l-1}k_{ij}^{l}+b_{j}^{l}\right). \end{array}$$

If there are *N* input images in the product layer, then the corresponding down-sampling layer also has *N* output images, but each output image is reduced compared to the original one. The formula is

(16) $$\begin{array}{c} x_{j}^{l}=f\left(\beta_{j}^{l}\text{down}\left(x_{j}^{l-1}\right)+b_{j}^{l}\right). \end{array}$$

First, sample the feature map of the *n* + 1 layer, and then calculate the sensitivity. The formula is

(17) $$\begin{array}{c} \delta_{j}^{l}=\beta_{j}^{l+1}\left(f^{\prime }\left(u_{j}^{l}\right)*\text{up}\left(\delta_{j}^{l+1}\right)\right). \end{array}$$

Among them, *∗* means dot multiplication, that is, multiplying each pixel, which represents an upsampling process. The process is as follows: the sampling factor is set to *n*, and then each element of the input layer is repeated horizontally and vertically, and the number of repetitions is *n* times; the formula is

(18) $$\begin{array}{c} \text{up}\left(x\right)=x⊗l_{n*n}. \end{array}$$

The sensitivity of the pixel is calculated by the sensitivity and classified according to the polynomial derivation rule. The formula is

(19) $$\begin{array}{c} \frac{\partial E}{\partial b_{j}}=\sum_{u,v}{\left(\delta_{j}^{l}\right)}_{uv}. \end{array}$$

For the convolution kernel, the backpropagation algorithm is used for processing, that is, the gradient of the convolution kernel corresponding to the feature map is

(20) $$\begin{array}{c} \frac{\partial E}{\partial k_{ij}^{l}}=\sum_{u,v}{\left(\delta_{j}^{l}\right)}_{uv}{\left(P_{i}^{l-1}\right)}_{uv}. \end{array}$$

Sample the feature maps for the *n*-layer and *n* − 1 layer, perform different assignments on the *n*-layer and *n* − 1 layer, and perform the partial derivative calculation; then, the partial derivative is

(21) $$\begin{array}{c} C_{1}\times S\left(\begin{array}{cc} 1 & 2\\ 4 & 5 \end{array}\right)+C_{2}\times S\left(\begin{array}{cc} 2 & 3\\ 5 & 6 \end{array}\right)+C_{3}\times S\left(\begin{array}{cc} 4 & 5\\ 7 & 8 \end{array}\right)+C_{4}\times S\left(\begin{array}{cc} 5 & 6\\ 8 & 9 \end{array}\right). \end{array}$$

After a simple verification, it can be written as the following formula:

(22) $$\begin{array}{c} \frac{\partial E}{\partial k_{ij}^{l}}=\text{rot}180\left(\text{conv}2\left(x_{i}^{l-1}\right.,\text{rot}180\left(\delta_{j}^{l}\right)\prime ,\text{valid}\prime \right). \end{array}$$

Then, the calculation result of the convolutional layer *C* is as follows (the convolution operation needs to first rotate the convolution kernel by 180 degrees and then perform related operations on the corresponding items).

(23) $$\begin{array}{c} C_{1}=S_{1}K_{1}+S_{2}K_{2}+S_{4}K_{3}+S_{5}K_{4},\\ C_{2}=S_{2}K_{1}+S_{3}K_{2}+S_{5}K_{3}+S_{6}K_{4},\\ C_{3}=S_{4}K_{1}+S_{5}K_{2}+S_{7}K_{3}+S_{8}K_{4},\\ C_{4}=S_{5}K_{1}+S_{6}K_{2}+S_{8}K_{3}+S_{9}K_{4}. \end{array}$$

When calculating the sensitivity of the corresponding convolutional layer, you need to use all the sensitivities associated with it, as follows:

(24) $$\begin{array}{c} C_{1}=S_{1}K_{1}+S_{2}K_{2}+S_{4}K_{3}+S_{5}K_{4},\\ C_{2}=S_{2}K_{1}+S_{3}K_{2}+S_{5}K_{3}+S_{6}K_{4},\\ C_{3}=S_{4}K_{1}+S_{5}K_{2}+S_{7}K_{3}+S_{8}K_{4},\\ C_{4}=S_{5}K_{1}+S_{6}K_{2}+S_{8}K_{3}+S_{9}K_{4}. \end{array}$$

When calculating the sensitivity of the *C* layer, it is necessary to use all the sensitivities related to it, which is

(25) $$\begin{array}{c} C_{1}=S_{1}K_{1}+S_{2}K_{2}+S_{4}K_{3}+S_{5}K_{4},\\ C_{2}=S_{2}K_{1}+S_{3}K_{2}+S_{5}K_{3}+S_{6}K_{4},\\ C_{3}=S_{4}K_{1}+S_{5}K_{2}+S_{7}K_{3}+S_{8}K_{4},\\ C_{4}=S_{5}K_{1}+S_{6}K_{2}+S_{8}K_{3}+S_{9}K_{4}. \end{array}$$

## 4. Teaching Promotion Platform

As the name implies, the online teaching platform is a distance teaching activity based on the Internet. From the concept of online teaching platform to the present, after many years of improvement and development, the online teaching system has gradually matured and achieved outstanding results in theory and practical applications. Not only that but also widely praised by people. From a global perspective, the widely used and more mature online teaching systems mainly include the Blackboard system and the WebCT system. The functions of the Blackboard system can be summarized in terms of inclusiveness and flexibility. It is embodied in the fact that it covers almost all the functions required for online teaching and can fully meet the needs of teachers using online teaching platforms. Flexibility is reflected in the strong functional scalability of the Blackboard system. It can increase system functions by changing the plug-in form to meet the needs of users according to changes in external needs. These two functional characteristics of the Blackboard system make the system widely used in almost every country in the world. Not only that, the system adopts a folder management mode for the management of teaching content and the operating system. This design is more in line with the daily life of users. Operating habits: the WebCT system was developed earlier than the Blackboard system, so it will take longer to develop and update. The system is developed on the basis of a web browser to realize the management of the entire online teaching process and the production and release of teaching resources. The main characteristics of the WebCT system can be summarized from two aspects: the first aspect is that the system can control the online teaching process, and the second aspect is the ability to make and publish teaching resources.

### 4.1. Online Teaching CSAL Platform System Demand Function Analysis

#### 4.1.1. Use Case Analysis of Teacher Participants

Teachers are the main participants in the traditional teaching mode, and they are an indispensable part in the online teaching CASL platform system. The online teaching mode is divided into two aspects: “teaching” and “learning.” Teachers solved the doubts by preaching. So, teachers are the main part of “teaching.” Teachers' main job in “teaching” is to design the process of online teaching, combining the characteristics of the learning content taught in their daily learning life and their own years of education and teaching experience, and arrange the teaching content and schedule correctly and reasonably, so that students can learn. Complete learning tasks efficiently and with high quality, and achieve a multiplier learning effect. Teacher participants' feedback on the system is more objective. They mainly hope that the online teaching system can meet the following four aspects: first, the teacher participants hope that the online teaching system can have the function of designing the teaching process and be able to bind relevant teaching resources, setting different transfer conditions, and other methods to realize the automatic jump of the process according to the actual learning situation of different students; second, teacher participants hope that the online learning system can perform real-time learning behaviors and activities of each student according to certain rules. Through the program, teachers can collect, observe, and analyze a large number of students' learning behavior data, as well as the homework, accuracy, examination results, and other data, so as to comprehensively and objectively understand and master each student's learning situation and learning process. Third, the teacher participants hope that the online learning system can create an intelligent auxiliary education environment, which can automatically classify and summarize the questions asked by students and at the same time classify all questions according to the number of questions. Questions are sorted so that teachers can focus on answering students' questions, and it is also helpful for teachers to discover and modify the deficiencies in teaching content in time so that online learning can achieve the best results; fourth, teacher participants hope that the online learning system can intelligently formulate scalable and repeatable online learning strategies and can formulate different learning strategies suitable for each student according to their different actual learning conditions, and supervise and feed back the learning conditions at the same time. Teacher use case design is shown in Figure 4.

#### 4.1.2. Use Case Analysis of Student Participants

Student participants are also important participants in the online learning platform system and are the main part of “learning” in the online teaching process. The main purpose of student participants using the online learning system is to conduct self-learning based on the teaching content formulated by the teacher and the teaching task as the goal. At the same time, to formulate a reasonable and effective learning task arrangement according to their characteristics and to use online learning shared teaching resources are used to complete the learning tasks. At the same time, in the process of independent learning, you can communicate and discuss with other students about learning. If you do not understand, you can ask the teacher in time. Leave any doubts and promote your understanding and mastery of the learning content. The feedback of student participants on the online learning system is more intuitive and specific than that of teacher participants. They hope that the online learning system can meet the following four aspects: first, student participants hope that the online learning system can learn through real-life examples providing process-oriented effective guidance so that students of various types can complete the assigned learning tasks by the correct learning steps under the guidance of the learning activities set in the entire process. Second, learning participants hope that the online learning system can automatically adjust the teaching methods and content based on the learning knowledge that students understand and master at this stage, realize intelligent learning supervision, and improve the learning ability and learning effect of students more rationally and effectively. Third, student participants hope that the online learning system can provide a supervising chat room or discussion area, which can record the effective time of each student's participation in the discussion, the number of speeches, the amount of speech, and other information and at the same time can provide information to the students. The discussed learning content is managed and supervised, and measures are taken for students who do not meet the requirements according to corresponding rules; fourth, student participants hope that the online learning system can record and monitor the learning situation of students in their daily learning life, and data analysis is carried out through the system rules and students' usual learning situation, and the problems existing in the learning process of students can be reflected and dealt with promptly. At the same time, the data recorded by the online learning system can be used as the basis for the final assessment. Student use case design is shown in Figure 5.

### 4.2. Principles of System Design

The design and development of the CSAL system is based on WF. The main purpose is to solve a series of problems in the current online teaching process, such as the lack of correct guidance for students' independent learning and teachers' inability to fully understand the students' learning level. In the process of design and development of the system, the following two basic development principles need to be followed: the first is the principle of modularization. In the process of designing the self-learning online teaching system, there are many general functional modules, such as access to the database, network communication support platform, and user management. These modules also exist in other information management systems and have more mature solutions, which allows the system to use existing resources to reduce workload during the design and development of the system. Not only that, the use of mature modules also contributes to the overall stability of the system. The second is the principle of advanced thinking and technology. At this stage, the research on workflow-related technologies has become more mature. However, the application of workflow technology in the field of autonomous learning platforms is still very rare. But in terms of theory and application process effect, workflow technology is completely suitable for online teaching systems. Therefore, it is necessary to be advanced in thinking and combine the workflow technology with the online teaching process of self-learning to create the core of the online teaching self-learning platform.

### 4.3. System Network Architecture Design

The system network architecture design is to design the network topology of the system deployment. The network architecture design is shown in Figure 6.

According to the above picture, we can find that the CSAL system is composed of the internal network and the external network. The internal network mainly provides server terminal services, and the external network mainly provides network services to users. In the internal network, the server is composed of the server component of the deployment system, the data storage server, and the application component of the deployment website. The external network adopts the B/S mode, and the server designed through the B/S mode is more convenient in the use process.

### 4.4. System Database Design

The teacher information data table mainly stores the basic information of the teachers in online teaching. The specific design is shown in Table 2.

The student information data table mainly stores relevant information data of student participants in the online teaching process. Student information data is shown in Table 3.

The learning resource data table records the learning content assigned to different students. The specific data table structure of learning resource is shown in Table 4.

## 5. System Function Test

Starting from the test, this article introduces the test process and results of specific functional modules of the platform from two aspects of the test environment and test cases, to verify the usability of the online teaching practice platform.

The platform of this article is a web application based on the B/S structure. This test is mainly based on the general IaaS cloud platform, using the cloud host as the test server, and the deployment environment mainly includes the web container Jetty and the database MySQL. The specific test environment content is shown in Table 5.

The functional testing of the learning platform is based on the user's real-life application scenarios, using a black-box testing method to perform detailed testing on the functional modules of the online teaching practice platform, and the testing will cover every functional point.

According to the test case set and typical test cases, the overall verification of the functions of the online teaching practice platform has been completed. It can be seen from the test results that the platform meets the basic requirements of functional design, and the test results are in line with expectations.

## 6. Conclusion

With the continuous advancement of social technology, artificial intelligence technology is also constantly developing. Due to the complex and changeable facial expressions of people, this makes the professional knowledge involved in face recognition more complex, and the professional knowledge involved is broader. Under this situation, face recognition technology has been constantly updated and developed. Based on this, the face recognition solution proposed in this article also needs to be updated in real-time with the latest technology. To improve the accuracy of face recognition. In addition, there are various mobile terminal platforms in society, mainly Android, Windows, and Phone. In the research process of this paper, we mainly take Android and Windows as examples. However, it is not representative to study these operating systems only. Therefore, we need to update and upgrade the platform and technology applied in the later stage of research, so as to make face recognition more accurate and correct, and meet the needs of more platform users.

With the development of society, in the process of promoting Chinese in the world today, we need to refine the Chinese language so that the Chinese we spread can be accepted by more people. At the same time, we need to explore the Chinese culture in depth. In the process of dissemination, we not only promote Chinese but also promote Chinese culture. The promotion of Chinese covers a wide range of fields, and it almost includes many subjects related to the promotion of Chinese such as linguistics, pedagogy, and management. Through investigation and research on relevant documents, it is found that Chinese promotion is not just a person's work, it requires the joint efforts of the whole society. Only by gathering the power of the whole country can we promote Chinese throughout the world and make the whole world feel Chinese. The charm of culture: due to the limitation of the author's knowledge reserves and energy, as well as limited resources, this research will not be comprehensive and in-depth, and there will inevitably be mistakes and omissions, which will be left for later scholars to study and supplement.

Based on workflow technology, we observe and compare students' learning conditions through the platform, analyze students' learning goals, learning effects, learning emotions, and conflicts and conflicts generated in the process of cooperation and find and resolve them in time these questions. At the same time, the workflow collects and records the learning situation and learning data of students and automatically reminds and corrects various problems existing in the learning process of students.

## Figures and Tables

**Figure 1:** Principles of the natural language understanding model.

**Figure 2:** Multilayer feedforward neural network.

**Figure 3:** Convolutional neural network model.

**Figure 4:** Teacher use case design.

**Figure 5:** Student use case design.

**Figure 6:** Network architecture design.

**Table 1:** Classification of machine learning.

Classification	Name	Definition	Typical application
Learning mode	Supervised learning	Supervised learning refers to a process of changing the parameters of the sample classifier so that the sample can meet the corresponding performance requirements. Supervised learning is also called supervised training or learning with teachers. To put it simply, it is to use a certain learning strategy or learning method to build a model through a limited training data set that has been labeled to realize the labelling or mapping of new data.	Natural Language Processing, etc.
	Unsupervised learning	In our daily lives, there will always be a series of problems that it is difficult to manually label its categories due to lack of sufficient experience and knowledge, or the cost of manually labelling categories is too high. So, we hope to use machines to help us accomplish these tricky things. Therefore, it is possible to use unmarked limited data to describe the structure or law hidden in the unmarked data, thereby solving various problems.	Data mining, etc.
	Reinforcement learning	Reinforcement learning is also called competitive learning or reinforcement learning. It is a behaviour that uses agents to interact with the external environment to obtain rewards. In simple terms, it is the autonomous learning that the intelligent system maps from the environment to behaviour through its own experience.	Autonomous driving, go, etc.

Study method	Traditional machine learning	Traditional machine learning includes a very wide range, but it is inseparable from the core of traditional machine learning: starting from training samples, through the analysis of certain principles, the corresponding laws are found to complete the prediction of future data behaviors or trends.	Natural Language Processing, speech recognition
	Deep learning	Deep learning integrates low-level features into more abstract high-level features. It is also a learning method to build a deeper structural model.	Don't wait
	Transfer learning	Transfer learning is also a kind of machine learning method. It takes the development model of one task as the starting point and reuses it in the process of the development model of another task.	Image identification

Other common algorithms	Active learning	The corresponding samples are screened out through algorithms, and then the samples are labelled. This method improves the accuracy of the model.	Positioning based on sensor network

**Table 2:** Teacher information data sheet.

No.	Field name	Field type	Field length	Remarks
1	ID	Int	8	Teacher ID number
2	Name	nchar	10	Name
3	Birthday	Datetime	8	Birthday
4	Sex	nchar	4	Gender
5	Profession	nchar	50	Profession
6	Level	nchar	10	Job title
7	Educational	nchar	10	Education

**Table 3:** Student information data sheet.

No.	Field name	Field type	Field length	Remarks
1	ID	Int	8	Student ID number
2	Name	nchar	10	Name
3	Birthday	Datetime	8	Birthday
4	Sex	nchar	4	Gender
5	Profession	nchar	50	Profession
6	Inschool	Datetime	8	Enrollment date

**Table 4:** Learning resource data table.

No.	Field name	Field type	Field length	Remarks
1	ID	Int	8	Learning resource ID number
2	Level	Int	8	Resource level
3	Profession	nchar	16	Professional field
4	AttendesID	Int	8	Participant ID
5	Updatetime	Datetime	8	Update time
6	FilelD	Int	8	Learning resource index

**Table 5:** Test environment content.

Operating system	CentOS release 6.4
Java environment	JDK 1.8.0 91
Database	MySQL 5.1.73
Web server	Jetty 8.1.6
Browser	Chrome 69.0.3497.100 (64 bit)

## Data Availability

The data used to support the findings of this study are available from the corresponding author upon request.
